# Targeting miR-185-3p Inhibits Head and Neck Squamous Cell Carcinoma by Modulating RAB25

**DOI:** 10.3389/fonc.2021.721416

**Published:** 2021-11-15

**Authors:** Xueping Wang, Xiaoyuan Zhu, Yulin Zhao

**Affiliations:** Department of Otolaryngology, The First Affiliated Hospital of Zhengzhou University, Zhengzhou, China

**Keywords:** head and neck squamous cell carcinoma, exosome, miR-185-3p, RAB25, tumor growth

## Abstract

Cancer cell-derived exosomes regulate tumor growth and progression. However, the effects of exosomes and its contents on head and neck squamous cell carcinoma (HNSCC) and its underlying mechanisms remain unclear. Here, we found HNSCC displayed a dysregulation of exosomes biogenesis. miR-185-3p was one of the most upregulated exosome-derived miRNAs in HNSCC. Functional assay showed that RAB25 is a direct downstream target of miR-185-3p. miR-185-3p/RAB25 signaling controlled tumor progression and correlated with disease prognosis. Targeting miR-185-3p/RAB25 significantly inhibited tumor growth and promoted drug response to chemotherapy. To conclude, the findings demonstrate exosomal miR-185-3p promotes tumor growth by mediating RAB25 that could be effectively targeted for HNSCC treatment.

## Introduction

Head and neck squamous cell carcinoma (HNSCC), including the squamous cell carcinoma of oral cavity, larynx, oropharynx, and hypopharynx, is a major frequently lethal malignancy with a yearly mortality of 40–50% (1, 2). Development of HNSCC is associated with the factors such as tobacco, alcohol consumption, human papillomavirus (HPV) infection, and TP53 mutation (3). Patients with HNSCC are commonly diagnosed at a progressed stage, and with unfavorable prognosis. Despite advances on therapies, such as radiotherapy, chemotherapy, immunotherapy, and their combination, the prognosis of HNSCC is dismal, and the survival time has not been greatly improved (4, 5). Therefore, exploring the potential mechanism of HNSCC prognosis and finding the relevant biomarkers that are responsible for the tumor progression and poor outcomes would be greatly imperative.

Intracellular communication is essential to the functional integrity of multicellular organisms. Exosomes, a kind of extracellular vesicles that formed by the inward budding or shedding from parent cells, has recently captured attention in cellular communication study (6). It has been demonstrated that exosomes mediate the crosstalk between cells and contribute to the interaction with cellular microenvironment and functional reprogramming by carrying biological contents from donor to target cells under both physiological and pathological conditions (7, 8). Tumor-derived exosomes were reported to accelerate tumor metastasis in several malignancies including HNSCC by releasing miRNAs (9). Exosomal miRNAs are suggested to modulate the behaviors of recipient cells by coordinating gene expression (10). Tumor cell-derived exosomal miR-21 promotes metastatic behaviors in oral squamous cell carcinoma cells, identified as the potential target for cancer therapy (11). miR-9-enriched exosomes from HNSCC increase the HNSCC radiosensitivity by polarizing macrophages into M1 phenotype (12). Moreover, multiple exosome-derived miRNAs have been identified as the biomarkers for diseases diagnosis owing to the high stability of exosomal miRNAs (13).

Rab25 belongs to Rab-GTPase family, in which protein dysregulation causes various pathophysiological diseases including cancer. Rab25 has diverse roles in the various types of cancers and functions as oncoprotein in bladder cancer, gastric cancer, lung cancer, whereas acts as tumor-suppressive protein in head and neck cancer, esophageal cancer, triple-negative breast cancer (14). Rab25 was regulated by different miRNAs in cancer progression, suggesting a possible miRNA-mediated mechanism in tumor biology (15, 16). The mechanisms underlying the difference in mediating diverse cancer types have not been fully defined.

In this study, we explored the role of tumor cell-derived exosomes in HNSCC, and further investigated the role of exosomal miRNAs on tumor behavior, as well as the involved molecular mechanisms.

## Materials and Methods

### Patients and Tissue Collection

A total of 31 HNSCC patients including eight classical (CL), ten basal (BA), seven mesenchymal (MS), and six atypical (AT) cases were randomly enrolled in the present study, who were firstly diagnosed at the First Affiliated Hospital of Zhengzhou University based on histopathological evaluation. Patients with histologically squamous cell carcinoma of the oral oropharynx were included. Patients who received preoperative radiotherapy, chemotherapy, or immunotherapy before the surgery were excluded. The 31 tumor tissues and 10 normal nasopharynx tissues were collected in the process of the surgery or biopsy. All tissue samples were immediately frozen in liquid nitrogen and stored at −80°C until required. All procedures performed in this study were in accordance with the ethical standards of the Ethics Committee of the First Affiliated Hospital of Zhengzhou University. The written informed consent was obtained from all participants prior to the sample collection.

### Real-Time PCR

Total RNA was extracted from cells using TRIzol reagent (Invitrogen), and RNA concentration was determined using NanoDrop-1000 spectrophotometer (Thermo Fisher Scientific). The isolated RNA was reversely transcribed into cDNA with primers (Sangon Biotech, Shanghai) using high-capacity RNA-to-cDNA kit (4368814, Applied Biosystems). For miRNA expression, exosomal miRNAs were isolated by using the SeraMir Exosome RNA Purification Kit (RA806A-1, System Biosciences, USA), and cDNA for miRNAs was synthesized using 1 μg of total RNA treated with DNase I and TaqMan microRNA assay kit (4427975, Applied Biosystems) as described in the manufacturer’s protocol. The qRT-PCR was conducted with the ABI Prism 7500 System using microRNA detection kit (Q32882, Thermo Fisher Scientific). Relative mRNA and miRNA expression were calculated using 2^−ΔΔCt^ method. The experiments were replicated in triplicate.

### Cell Culture and Transfection

Human oral squamous cell carcinoma cell lines HN4 and HN6 and normal nasopharyngeal epithelial cells NP69 were from Cell Bank of the Chinese Scientific Academy. All cells were grown in RPMI 1640 medium supplemented with 10% fetal bovine serum (FBS) and 1% penicillin/streptomycin (Invitrogen) in a humidified incubator at 37°C with 5% CO_2_ and 95% air. For cell transfection, shRNA targeting CD63, TSG101 (Horizon, CA, USA), the siRNA targeting miR-185-3p, pcDNA containing miR-185-3p, and their control DNA (OriGene, MD, USA) were conducted using Lipofectamine™ 2000 (Thermo Fisher Scientific, USA) according to the manufacturer’s instructions.

### Western Blot

Cells were lysed using RIPA buffer (Beyotime, China), quantified by BCA protein assay kit (Beyotime, China), subjected to a 10% sodium dodecyl sulfate polyacrylamide gel (SDS-PAGE) for electrophoresis, and subsequently transferred onto a polyvinylidene difluoride membrane (PVDF). The membrane was incubated with primary antibodies RAB25 (4314, Cell Signaling), CD63 (ab134045, Abcam), CD9 (13409, Cell Signaling), TSG101 (ab133586, Abcam), or Calnexin (2433, Cell Signaling) at 4°C overnight, followed by incubation with peroxidase-linked secondary antibodies (ab6721, Abcam) for 1 h at RT. The bands were visualized using an enhanced chemiluminescence reagent (Thermo Fisher Scientific, USA). The relative protein expression was normalized to GAPDH.

### Dual-Luciferase Reporter Assays

The experiment was conducted using the dual-luciferase reporter assays according to the instruction (Promega Corporation, Madison, WI, USA). Briefly, the sequences of wildtype (WT) RAB25 3’-UTR (wild-type 3’-UTR) reporter plasmids and the mutant one (Mut) mapping the miR-185-3p-binding site were conducted using Site-directed mutagenesis. The WT or Mut RAB25 was cloned into the psiCHECK-2 vector for luciferase reporter assays. The vector was co-transfected with miR-185-3p mimics or the control sequence into HN4 and HN6 cells using the Dual-Luciferase Reporter Assay System (Promega Corporation, Madison, WI, USA), and firefly luciferase activity was measured by Reporter Assay System Kit (Promega) at 24 h after transfection.

### Cell Viability and Colony Formation

Cell viability was measured using MTT assays (Beyotime, Shanghai, China). Briefly, Cells were placed in a 96-well plate at a density of 2,000 cell/well to allow cell adherence. After incubating with 15 μl MTT solution (5 mg/ml) (Sigma-Aldrich, MO, USA) in each well for 4 h, the absorbance was measured under the wavelength of 570 nm using a microplate reader. Cells were plated in a six-well plate at a density of 300 cells per well and culture in the colony forming medium (Sigma-Aldrich, USA). After culture, cells were fixed using 4% paraformaldehyde for 15 min and washed with PBS. The colonies were stained with 0.1% crystal violet staining solution for 30 min and finally calculated using ImageJ software.

### Exosome Isolation

Exosome isolation was conducted according to the MISEV 2018 guidelines. Briefly, after cells culture for about 48 h and reaching 80% confluence, the cultured cells and medium were collected for ultrafiltration with 2,000 g for 30 min to remove cells and debris. The supernatant was filtered through 0.22 μm filters (Merck Millipore) and transferred into a new tube with the addition of the total exosome isolation reagent for incubation at 4°C overnight. After incubation, the samples were ultracentrifuged at 100,000 × g for 1 h at 4°C. Exosomes in the pellet at the bottom of the tube were collected and resuspend in 1× PBS, followed by a second round of ultracentrifugation. The obtained exosomes were purified using an OptiPrep™ density gradient according to manufacturer’s instruction (D1556, Sigma Aldrich), and were characterized and quantified using Western blot, Transmission Electron Microscope (TEM), and nanoparticle tracking analysis (NTA).

### *In Vivo* Tumorigenesis

Six-to-eight-week-old NOD/SCID mice were purchased from Shanghai Lab. Animal Research Center (Shanghai, China), and housed in the ventilated cage under condition of 25°C, with 70% humidified air. All mice were kept at a 12 h light/night cycle for 1 week before the experiment. The animal experiments were conducted by the approval of the Ethics Committee at the First Affiliated Hospital of Zhengzhou University. The animal use and care were in accordance with the guidelines of this committee. For tumor formation assay, 1×10^5^ HN4 cells with miR-185-3p overexpress or its negative control were suspended in 100 μl PBS and subcutaneously injected into the mice. Tumor volumes were monitored once a week for 4 weeks. For drug response assay, HN4 cells were subcutaneously injected into NOD/SCID mice to form tumor burden. Tumor-bearing NOD/SCID mice were then intravenously injected with 10 mg/kg docetaxel (2 mg/ml dissolved in 0.9% saline), miR-185-3p inhibitor, 10 mg/kg docetaxel+ miR-185-3p inhibitor, or the same volume of saline every 2 days for 6 days. Tumor size was monitored for the next 30 days. Mice with a significant tumor shrinkage after drug administration was defined as response to treatment compared to control group.

### RNA Sequencing and Data Analysis

For RNA sequencing assay, total RNA was isolated from tumor and normal tissues and subjected to the subsequent RNA sequencing at Beijing Genomics Institute (BGI, Shenzhen, China). Differentially expressed genes (DEGs) were analyzed by using edgeR package in R. Gene ontology (GO) analysis was performed based on the DEGs using DAVID 6.7. A *p*-value <0.01 denoted significant enrichments in the GO pathways. For TCGA analysis, the expression and survival rate as well as the correlation of miR-185-3p and RAB25 were investigated in HNSCC using the online TCGA data by the tool UALCAN (http://ualcan.path.uab.edu/index.html).

### Statistical Analysis

Data were presented as means ± SD. GraphPad Prism 7 software was conducted to analyze statistics. Unpaired t-test was performed to analyze the differences between two groups, while one-way ANOVA followed by Holm-Oak’s multiple comparisons were conducted to compare the difference among more than two groups. A value of p < 0.05 was considered significant.

## Results

### Exosome Biogenesis Is Upregulated in HNSCC

To investigate the regulating mechanism of HNSCC progression, we firstly performed mRNA sequencing on HNSCC tumor tissues (n=31) and normal nasopharynx tissues (n=10) to uncover the differentially expressed genes (DEGs) in HNSCC. Compared with the normal tissues, we found a remarkable difference of gene expression profiles in between tumor and normal tissues (**Figure 1A**, Fold-change>2.0, *p*<0.01). Pathway analysis showed that those DEGs were associated with retinol dehydrogenase activity, extracellular space, and especially extracellular exosome (**Figure 1B**), suggesting exosome biogenesis/secretion was dysregulated in HNSCC. Next, we confirmed a significant elevation of mRNA expressions of exosomal markers TSG101 and CD63 in cell lines HN4 and HN6 compared with normal cell lines NP69 (**Figures 1C, D**). Moreover, exosome numbers increased in HN4 and HN6 compared with NP69 (**Figure 1E**). The data indicated that exosome biogenesis was upregulated in HNSCC.

**Figure 1:** Exosome biogenesis is upregulated in HNSCC. **(A)** Heatmap shows the expression profile of differentially expressed genes between HNSCC tumor tissues and Normal tissues. **(B)** Enrichment pathway analysis was performed to analyze the dysregulated pathways. **(C, D)** TSG101 and CD63 mRNA expression in HN4, HN6, and NP69. **(E)** The exosome number in NP69 and HNSCC cell lines HN4 and HN6. All experiments were replicated in triplicate. *p < 0.05.

### A Changed miRNAs Expression Profile in HNSCC Cell-Derived Exosomes

Exosomes contain a set of functional nucleic acids and are the main source of circulating miRNAs (17). Next, we performed miRNA sequencing on exosomes from HN4 and NP69. We found many miRNAs were dysregulated in HN4 compared with NP69 (**Figure 2A**). And miR-185-3p was one of the most five upregulated miRNAs (**Figure 2B**). qRT-PCR confirmed tumor cells expressed increased level of miR-185-3p compared with NP69 (**Figure 2C**). To verify the effects of exosome biogenesis on miR-185-3p level, we performed shRNA specifically targeting CD63 or TSG101 and detected the changes of exosome numbers and miR-185-3p expression. It showed that knockdown of CD63 (shCD63) or TSG101 (shTSG101) significantly resulted in decreased exosome number and miR-185-3p expression (**Figures 2D, E**). The results showed that exosomes from HNSCC cells had changed expression profiles of the contained miRNAs.

**Figure 2:** A changed miRNAs expression profile in HNSCC cells-derived exosomes. **(A)** Volcano plot shows the dysregulated miRNAs in tumor-derived exosomes compared with normal ones. **(B)** Expressions of the most dysregulated miRNAs in exosomes of HN4 cells confirmed by qRT-PCR. **(C)** The expressions of miR-185-3p expression in HN4, HN6, and NP69. **(D)** Exosome numbers in cells with shCD63 or shTSG101 knockdown or control ones. **(E)** miR-185-3p expression in both HN4 and NH6 cells with shCD63 or shTSG101 knockdown or control ones. All experiments were replicated in triplicate. *p < 0.05.

### RAB25 Is a Direct Target of miR-185-3p

Next, we investigated the potential biological effects of exosome-contained miR-185-3p on HNSCC. The potential downstream targets of miR-185-3p were predicted using online TargetScan, and RAB25 is the most potential target of miR-185-3p. Subsequently, we confirmed the relationship between miR-185-3p and RAB25 using qRT-PCR and Western blot. It exhibited that miR-185-3p knockdown enhanced RAB25 expression (**Figures 3A, C**), and miR-185-3p overexpression decreased RAB25 expression at transcriptional and translational level (**Figures 3B, C**). Moreover, dual-luciferase reporter assay confirmed that overexpression of miR-185-3p significantly suppressed the luciferase activity in wild-type of RAB25, but not the mutant one (**Figures 3D, E**). The data indicated that RAB25 was a direct downstream target of miR-185-3p.

**Figure 3:** RAB25 is a direct target of miR-185-3p. **(A)** The mRNA expression of RAB25 in HN4 and HN6 cells with miR-185-3p knockdown. **(B)** The mRNA expression of RAB25 in HN4 and HN6 cells with miR-185-3p overexpression. **(C)** The expression of RAB25 protein in HN4 and HN6 cells with miR-185-3p knockdown or miR-185-3p overexpression. **(D)** graphic illustration showing the miR-185-3p binding site of RAB25 3’UTR as well as the mutate site. **(E)** Luciferase activity in HN4 and HN6 cells with WT or mutated miR-185-3p binding site. All experiments were replicated in triplicate. **p < 0.01, ***p < 0.001.

### miR-185-3p/RAB25 Mediates Tumor Cell Proliferation and Colony Formation

RAB25, a member of the Rab11 small GTPase family, mediates cancer progression, and is downregulated in oral and oropharyngeal squamous cell carcinoma (18). Subsequently, we investigated the effects of miR-185-3p/RAB25 on cell viability and colony formation in HN4 cells. miR-185-3p knockdown or RAB25 overexpression inhibited cell viability and colony formation (**Figures 4A–D**). Conversely, RAB25 overexpression also reversed miR-185-3p-promoted cell viability and colony formation compared with the control cells (**Figures 4E, F**). Both RAB25 overexpression and miR-185-3p knockdown remarkably inhibited cell viability and colony formation (**Figures 4G, H**), suggesting potential antitumor effects by targeting miR-185-3p/RAB25.

**Figure 4:** miR-185-3p/RAB25 mediates tumor cell proliferation and colony formation. **(A)** Cell viability of HN4 with miR-185-3p knockdown or WT HN4 cells. **(B)** Cell colony number of HN4 with miR-185-3p knockdown or WT HN4 cells. **(C)** Cell viability of HN4 with RAB25 overexpression or WT HN4 cells. **(D)** Cell colony number of HN4 with RAB25 overexpression or WT HN4 cells. **(E)** Cell viability of HN4 with miR-185-3p overexpression, miR-185-3p/RAB25 overexpression, or WT HN4 cells. **(F)** Cell colony number of HN4 with miR-185-3p overexpression, miR-185-3p/RAB25 overexpression, or WT HN4 cells. **(G)** Cell viability of HN4 with miR-185-3p knockdown, miR-185-3p knockdown/RAB25 overexpression, or WT HN4 cells. **(H)** Cell colony number of HN4 with miR-185-3p knockdown, miR-185-3p knockdown/RAB25 overexpression, or WT HN4 cells. All experiments were replicated in triplicate. *p < 0.05.

### miR-185-3p/RAB25 Is Deregulated and Associated With Poor Prognosis in HNSCC

Next, the expression levels of miR-185-3p and RAB25 in HNSCC tumor tissues were investigated using qRT-PCR. miR-185-3p expression was remarkably increased in tumor tissues compared with the normal (**Figure 5A**). Conversely, RAB25 levels were remarkably reduced in tumor tissues compared with the normal (**Figure 5B**). TCGA analysis demonstrated HNSCC patients exhibited higher expression of miR-185-3p and lower expression of RAB25 as compared with normal individuals (**Figures 5C, D**). The expression of miR-185-3p and RAB25 were also correlated with tumor grade and nodal metastasis stratification (**Figures 5E–H**). High miR-185-3p expression correlated with lower survival rate in HNSCC patients (**Figure 5I**), which is not significantly different in patients with different expression of RAB25 (**Figure 5J**). The data demonstrated that the miR-185-3p/RAB25 was deregulated and associated with poor prognosis in HNSCC.

**Figure 5:** miR-185-3p/RAB25 is deregulated and associated with poor prognosis in HNSCC. **(A, B)** mRNA expression of miR-185-3p and RAB25 in HNSCC tumor and adjacent tissues. **(C, D)** TCGA data showing the relative expression of miR-185-3p and RAB25 in HNSCC patients and normal ones. **(E, F)** TCGA data showing the relative expression of miR-185-3p and RAB25 in HNSCC patients with different node metastasis stratification. **(G, H)** TCGA data showing the relative expression of miR-185-3p and RAB25 in HNSCC patients with different disease grade. **(I, J)** TCGA data showing the survival rate of miR-185-3p and RAB25 in HNSCC patients with different expression. *p < 0.05.

### Targeting miR-185-3p/RAB25 Therapeutically Inhibits Cancer Progression

To determine the role of miR-185-3p/RAB25 in tumor formation *in vivo*, cells were overexpressed with miR-185-3p or knocked down of RAB25 and then subcutaneously injected into the mice, respectively. It demonstrated that overexpression of miR-185-3p or knockdown of RAB25 increased tumor growth *in vivo* (**Figures 6A, B**). Next, we investigated its therapeutic effects by using miR-185-3p inhibitor. Mice were subcutaneously injected with tumor cells to form tumor burden, and then followed by treatment with miR-185-3p inhibitor. Chemical drug docetaxel was used as the parallel control. We found that miR-185-3p inhibitor significantly decreased the tumor progression *in vivo* (**Figure 6C**), as four of six mice exhibited stable or constrained tumor progression in miR-185-3p inhibitor-treated group; five of six mice exhibited stable or constrained tumor progression in docetaxel-treated group. Moreover, combined treatment of docetaxel and miR-185-3p inhibitor exhibited more effective on tumor inhibition *in vivo*, as all six mice responded to treatment strategy (**Figure 6C**). IHC also showed an increased level of RAB25 expression in tumor tissues of miR-185-3p inhibitor-treated and combination treatment groups (**Figure 6D**), confirming the anti-tumor effects of miR-185-3p inhibitor. The results uncovered a therapeutic role of miR-185-3p/RAB25 for HNSCC treatment.

**Figure 6:** Targeting miR-185-3p/RAB25 therapeutically inhibits cancer progression. **(A, B)** Tumor volume of mice injected with HN4 with miR-185-3p overexpression or RAB25 knockdown (n=6). **(C)** The drug response was monitored by evaluating the change of tumor size in tumor-bearing mice after administration with miR-185-3p inhibitor, docetaxel, or combination therapy (n=6). **(D)** Quantification and IHC images show the RAB25 expression in tumor tissue of different mice in **(C)**, *p < 0.05.

## Discussion

Exosome-derived miRNAs modulate the function of recipient cells, and (19) could be used for cancer diagnosis and treatment (19). Our present study found tumor-derived exosomes carried abundant miR-185-3p and promoted increased cell viability and colony formation ability. miR-185-3p was significantly increased in the HNSCC cells and tissues and had a binding site with the 3’UTR of RAB25. Therefore, we inferred that the aberrant expression of RAB25 is regulated by miR-185-3p that promotes HNSCC progression.

Exosomes were found to secrete externally by cells and ubiquitously exist in the body fluids, which makes it possible that exosomes could be taken as the biomarkers or targets for early diagnosis and therapy (20). Therefore, we focused on the role of tumor-derived exosomes on HNSCC, and to thoroughly study the intercellular crosstalk between exosomes and tumor cells. In the current study, we found exosome biogenesis was upregulated in HNSCC, which suggests exosomes may be associated with the pathogenesis of HNSCC. Exosomes could influence the tumor pathogenesis by interacting with the recipient cells, among which the content of exosomes, such as proteins, DNAs, metabolites, and RNAs, modulating cellular microenvironments (8). Mature miRNAs within exosomes were delivered to recipient cells, thereby regulating multiple processes by regulating gene expression, consequently influencing the function of recipient cells (21). In the present study, miR-185-3p, as a functional cargo miRNA within the HNSCC cells-derived exosomes, was increased and therefore regulating the expression of RAB25, suggesting miR-185-3p/RAB25 signaling serves as novel target for HNSCC treatment.

Tumor progression is connected with the development of drug resistance (22). Small guanosine triphosphates (GTPases) are the novel regulators on cancer development and progression (23). RAB25 is a small GTPases belongs to the member of RAB protein family and is a tumor suppressor in HNSCC (23, 24). It demonstrated that expression of RAB25 is associated with tumor progression, and loss of RAB25 leads to cell migration and invasion (25). Herein, we found that upregulated RAB25 decreased both cell proliferation and colony formation ability *in vitro*. Importantly, HNSCC mice showed more sensitivity to docetaxel when pretreated with miR-185-3p inhibitor, and overexpression of RAB25 blunted the effects of miR185-3p, indicating that the increased miR-185-3p promoted drug resistance by targeting RAB25.

In summary, our study identified the crucial role of tumor-derived exosomes and its packaged miRNAs on tumor progression, drug response. Importantly, we elucidated that tumor-derived exosomes-enriched miR-185-3p mediates tumor cell proliferation, colony formation, tumor growth, and drug response by targeting its downstream effector RAB25 that have potential therapeutic efficacy for HNSCC treatment.

## Data Availability Statement

The original contributions presented in the study are included in the article/supplementary material. Further inquiries can be directed to the corresponding author.

## Ethics Statement

All procedures performed in this study were in accordance with the ethical standards of the Ethics Committee of the First Affiliated Hospital of Zhengzhou University. The written informed consent was obtained from all participants prior to the sample collection.

## Author Contributions

XW and YZ conceived the study and drafted the manuscript. XW and XZ performed the experiments. XW contributed to the quality. All authors contributed to the article and approved the submitted version.

## Funding

This work was supported by the National Science Foundation (grant nos.82071023), the Henan Natural Science Foundation (grant nos. 202300410382), the Youth Foundation of The First affiliated Hospital of ZhengZhou University (no.YNQN2017001).

## Conflict of Interest

The authors declare that the research was conducted in the absence of any commercial or financial relationships that could be construed as a potential conflict of interest.

## Publisher’s Note

All claims expressed in this article are solely those of the authors and do not necessarily represent those of their affiliated organizations, or those of the publisher, the editors and the reviewers. Any product that may be evaluated in this article, or claim that may be made by its manufacturer, is not guaranteed or endorsed by the publisher.

## References

[1] FerlayJSoerjomataramIDikshitREserSMathersCRebeloM. Cancer Incidence and Mortality Worldwide: Sources, Methods and Major Patterns in GLOBOCAN 2012. Int J Cancer (2015) 136(5):E359–86. doi: 10.1002/ijc.29210 25220842

[2] BrayFFerlayJSoerjomataramISiegelRLTorreLAJemalA. Global Cancer Statistics 2018: GLOBOCAN Estimates of Incidence and Mortality Worldwide for 36 Cancers in 185 Countries. CA Cancer J Clin (2018) 68(6):394–424. doi: 10.3322/caac.21492 30207593

[3] CaponioVCATroianoGAdipietroIZhurakivskaKArenaCMangieriD. Computational Analysis of TP53 Mutational Landscape Unveils Key Prognostic Signatures and Distinct Pathobiological Pathways in Head and Neck Squamous Cell Cancer. Br J Cancer (2020) 123(8):1302–14. doi: 10.1038/s41416-020-0984-6 PMC755395732684626

[4] RaginCCModugnoFGollinSM. The Epidemiology and Risk Factors of Head and Neck Cancer: a Focus on Human Papillomavirus. J Dent Res (2007) 86(2):104–14. doi: 10.1177/154405910708600202 17251508

[5] Cancer Genome Atlas N. Comprehensive Genomic Characterization of Head and Neck Squamous Cell Carcinomas. Nature (2015) 517(7536):576–82. doi: 10.1038/nature14129 PMC431140525631445

[6] ClaytonABuschmannDByrdJBCarterDRFChengLComptonC. Summary of the ISEV Workshop on Extracellular Vesicles as Disease Biomarkers, Held in Birmingham, UK, During December 2017. J Extracell Vesicles (2018) 7(1):1473707. doi: 10.1080/20013078.2018.1473707 31162490PMC5965025

[7] NiuCWangXZhaoMCaiTLiuPLiJ. Macrophage Foam Cell-Derived Extracellular Vesicles Promote Vascular Smooth Muscle Cell Migration and Adhesion. J Am Heart Assoc (2016) 5(10):e004099. doi: 10.1161/JAHA.116.004099 27792649PMC5121506

[8] TheryCZitvogelLAmigorenaS. Exosomes: Composition, Biogenesis and Function. Nat Rev Immunol (2002) 2(8):569–79. doi: 10.1038/nri855 12154376

[9] XiaoCSongFZhengYLLvJWangQFXuN. Exosomes in Head and Neck Squamous Cell Carcinoma. Front Oncol (2019) 9:894. doi: 10.3389/fonc.2019.00894 31620359PMC6759986

[10] NguyenMAKarunakaranDGeoffrionMChengHSTandocKPerisic MaticL. Extracellular Vesicles Secreted by Atherogenic Macrophages Transfer MicroRNA to Inhibit Cell Migration. Arterioscler Thromb Vasc Biol (2018) 38(1):49–63. doi: 10.1161/ATVBAHA.117.309795 28882869PMC5884694

[11] LiLLiCWangSWangZJiangJWangW. Exosomes Derived From Hypoxic Oral Squamous Cell Carcinoma Cells Deliver miR-21 to Normoxic Cells to Elicit a Prometastatic Phenotype. Cancer Res (2016) 76(7):1770–80. doi: 10.1158/0008-5472.CAN-15-1625 26992424

[12] TongFMaoXZhangSXieHYanBWangB. HPV + HNSCC-Derived Exosomal miR-9 Induces Macrophage M1 Polarization and Increases Tumor Radiosensitivity. Cancer Lett (2020) 478:34–44. doi: 10.1016/j.canlet.2020.02.037 32120025

[13] SalehiMSharifiM. Exosomal miRNAs as Novel Cancer Biomarkers: Challenges and Opportunities. J Cell Physiol (2018) 233(9):6370–80. doi: 10.1002/jcp.26481 PMC1348244629323722

[14] AgarwalRJurisicaIMillsGBChengKW. The Emerging Role of the RAB25 Small GTPase in Cancer. Traffic (2009) 10(11):1561–8. doi: 10.1111/j.1600-0854.2009.00969.x PMC325849719719478

[15] YinCMouQPanXZhangGLiHSunY. MiR-577 Suppresses Epithelial-Mesenchymal Transition and Metastasis of Breast Cancer by Targeting Rab25. Thorac Cancer (2018) 9(4):472–9. doi: 10.1111/1759-7714.12612 PMC587905329524309

[16] XuPJiaSWangKFanZZhengHLvJ. MiR-140 Inhibits Classical Swine Fever Virus Replication by Targeting Rab25 in Swine Umbilical Vein Endothelial Cells. Virulence (2020) 11(1):260–9. doi: 10.1080/21505594.2020.1735051 PMC705114432114898

[17] SchwarzenbachHHoonDSPantelK. Cell-Free Nucleic Acids as Biomarkers in Cancer Patients. Nat Rev Cancer (2011) 11(6):426–37. doi: 10.1038/nrc3066 21562580

[18] ClausenMJMelchersLJMastikMFSlagter-MenkemaLGroenHJLaanBF. RAB25 Expression Is Epigenetically Downregulated in Oral and Oropharyngeal Squamous Cell Carcinoma With Lymph Node Metastasis. Epigenetics (2016) 11(9):653–63. doi: 10.1080/15592294.2016.1205176 PMC504871927379752

[19] HuYRaoSSWangZXCaoJTanYJLuoJ. Exosomes From Human Umbilical Cord Blood Accelerate Cutaneous Wound Healing Through miR-21-3p-Mediated Promotion of Angiogenesis and Fibroblast Function. Theranostics (2018) 8(1):169–84. doi: 10.7150/thno.21234 PMC574346729290800

[20] NamGHChoiYKimGBKimSKimSAKimIS. Emerging Prospects of Exosomes for Cancer Treatment: From Conventional Therapy to Immunotherapy. Adv Mater (2020) 32(51):e2002440. doi: 10.1002/adma.202002440 33015883

[21] JeffriesJZhouWHsuAYDengQ. miRNA-223 at the Crossroads of Inflammation and Cancer. Cancer Lett (2019) 451:136–41. doi: 10.1016/j.canlet.2019.02.051 PMC644162130878527

[22] HraskaVWoodsRK. Multiple Ventricular Septal Defects - Strategy, Sandwich, and Vanishing Bands. Semin Thorac Cardiovasc Surg (2019) 31(1):97–8. doi: 10.1053/j.semtcvs.2018.11.004 30447290

[23] TongMChanKWBaoJYWongKYChenJNKwanPS. Rab25 is a Tumor Suppressor Gene With Antiangiogenic and Anti-Invasive Activities in Esophageal Squamous Cell Carcinoma. Cancer Res (2012) 72(22):6024–35. doi: 10.1158/0008-5472.CAN-12-1269 22991305

[24] Tellez-GabrielMArroyo-SoleraILeonXGallardoALopezMCespedesMV. High RAB25 Expression Is Associated With Good Clinical Outcome in Patients With Locally Advanced Head and Neck Squamous Cell Carcinoma. Cancer Med (2013) 2(6):950–63. doi: 10.1002/cam4.153 PMC389240024403269

[25] AmornphimolthamPRechacheKThompsonJMasedunskasALeelahavanichkulKPatelV. Rab25 Regulates Invasion and Metastasis in Head and Neck Cancer. Clin Cancer Res (2013) 19(6):1375–88. doi: 10.1158/1078-0432.CCR-12-2858 PMC360223723340300

